The article "Intestinal fatty acid‐binding protein mediates atherosclerotic progress through increasing intestinal inflammation and permeability" was retracted in 2022. Reasons: duplicated images; signs of a paper mill.

# Intestinal fatty acid‐binding protein mediates atherosclerotic progress through increasing intestinal inflammation and permeability

**DOI:** 10.1111/jcmm.15173

**Published:** 2020-03-27

**Authors:** Lulu Zhang, Fan Wang, Jiajun Wang, Yongshun Wang, Yan Fang

**Affiliations:** ^1^ Department of Cardiology 2nd Affiliated Hospital of Harbin Medical University Harbin China; ^2^ The Key Laboratory of Myocardial Ischemia Harbin Medical University Ministry of Education Harbin China

**Keywords:** atherosclerosis, inflammation, intestinal fatty acid‐binding protein, intestinal permeability

## Abstract

Atherosclerosis is one of leading phenotypes of cardiovascular diseases, featured with increased vascular intima‐media thickness (IMT) and unstable plaques. The interaction between gastrointestinal system and cardiovascular homeostasis is emerging as a hot topic. Therefore, the present study aimed to explore the role of an intestinal protein, intestinal fatty acid‐binding protein (I‐FABP/FABP2) in the atherosclerotic progress. In western diet–fed ApoE^−/−^ mice, FABP2 was highly expressed in intestine. Silence of intestinal *Fabp2* attenuated western diet–induced atherosclerotic phenotypes, including decreasing toxic lipid accumulation, vascular fibrosis and inflammatory response. Mechanistically, intestinal *Fabp2* knockdown improved intestinal permeability through increasing the expression of tight junction proteins. Meanwhile, intestinal *Fabp2* knockdown mice exhibited down‐regulation of intestinal inflammation in western diet–fed ApoE^−/−^ mice. In clinical patients, the circulating level of FABP2 was obviously increased in patients with cardiovascular disease and positively correlated with the value of carotid intima‐media thickness, total cholesterol and triglyceride. In conclusion, FABP2‐induced intestinal permeability could address a potential role of gastrointestinal system in the development of atherosclerosis, and targeting on intestinal FABP2 might provide a therapeutic approach to protect against atherosclerosis.

## 1 INTRODUCTION

Atherosclerosis is one of leading causes of cardiovascular morbidity and mortality, including coronary heart disease, stroke and heart failure.^1^ Atherosclerosis cardiovascular diseases, featured with increased vascular intima‐media thickness (IMT) and unstable plaques, have multiple pathological signalling pathways.^1^ Excessive systemic and local inflammatory responses severely damage the vascular homeostasis. Emerging studies have found that endotoxin, mainly from gastrointestinal tissues, was linked to metabolic diseases and atherogenesis.^2^ Moreover, western diet increased plasma endotoxin activity in atherosclerotic patients, which could be attributed to the in intestinal disorders.^3^, ^4^ The intestine‐leaked endotoxins, such as lipopolysaccharide, was strong inflammatory stimuli in cardiovascular.^5^ Therefore, it is necessary to avoid the circulating toxic substances by manipulating the intestine‐cardiovascular interaction.

The article "Intestinal fatty acid‐binding protein mediates atherosclerotic progress through increasing intestinal inflammation and permeability" was retracted in 2022. Reasons: duplicated images; signs of a paper mill.

Intestinal permeability determines the circulating uptake of toxic substances and consequent cardiovascular diseases. In patients with chronic heart failure, their intestines exhibited injured gut mucosa and increased permeability.^6^, ^7^ Meanwhile, the circulating level of inflammatory tumour necrosis factor (TNF)‐α was significantly up‐regulated in these patients.^6^ Several animal studies have demonstrated that atherosclerotic mice had increased intestinal permeability, whereas improvement of intestinal permeability effectively suppressed atherosclerotic process.^5^, ^8^ Mechanistically, intestinal permeability was mainly regulated by intestinal epithelial zonulin proteins, such as zonula occludens 1 (ZO‐1) and occludin. Previous clinical study identified serum level of zonulin was closely related to circulating endotoxin concentrations in patients with myocardial infarction.^9^ Meanwhile, intestinal inflammation was one of key factors determining the biogenesis and function of epithelial zonulin proteins, and consequent the intestinal tight junction. In some autoimmune diseases, the tight junction integrity was severely disrupted by abnormal inflammatory response.^10^ Some beneficial intervention could protect against the intestinal inflammation‐induced disruption of tight junction.^11^, ^12^

Fatty acid‐binding proteins (FABPs), as lipid chaperones, mediate multiple lipid‐mediated biological processes and systemic metabolic homeostasis.^13^ Among them, FABP2, named intestinal FABP, is mainly expressed in intestinal epithelial cells. Patients with exercise training had higher plasma level of FABP2, which showed a positive correlation with gut permeability.^14^ FABP2 was considered as a biomarker of intestinal injury.^15^, ^16^ FABP2 was also involved in the inflammatory process. In patients with active ulcerative colitis, the plasma FABP2 level was obviously increased.^17^ The plasma FABP2 level was also up‐regulated in patients with acute intestinal ischaemia.^18^ However, it was unknown whether intestinal FABP2 could stimulate atherosclerotic progress through impairing intestinal permeability.

To address the role of intestinal FABP2 in atherosclerotic development, we specifically silenced intestinal *Fabp2* in high‐fat high‐cholesterol (HFHC) diet–fed ApoE‐deficient atherosclerotic mice. The present study supported the pathophysiological role of FABP2 in intestinal permeability and vascular homeostasis, and further modulated the development of atherosclerosis.

The article "Intestinal fatty acid‐binding protein mediates atherosclerotic progress through increasing intestinal inflammation and permeability" was retracted in 2022. Reasons: duplicated images; signs of a paper mill.

## 2 MATERIALS AND METHODS

### 2.1 Reagents

The haematoxylin (#MHS16) and eosin solution (#HT110116), Masson trichrome (#HT15) and Oil Red O (#3125‐12) staining kit were purchased from Sigma chemicals (Sigma). Anti‐FABP2 (#ab126744), anti‐moma‐2 (#ab33451) and anti‐α‐sma (#ab7817) antibodies were purchased from Abcam. Anti‐ZO‐1 (#13663), anti‐occludin (#91131) and anti‐Tubulin (#2146) antibodies were purchased from Cell Signaling. ELISA kits for measuring intestinal TNF‐α (#88‐7324‐22), IL‐1β (#88‐7013‐22) and MCP‐1 (#88‐7391‐22) levels were purchased from Invitrogen (Thermo Fisher). Biochemical kit for detecting endotoxin level and DX‐4000‐FITC reagent (#46944) were purchased from Sigma chemicals (Sigma, St. Louis). The lentivirus encoding *villin*‐drived *Fabp2* siRNA (#SASI_Mm01_00024824) was purchased from Sigma chemicals (Sigma).

### 2.2 Mouse experiment

Male ApoE knockout mice (ApoE^−/−^, purchased from Shanghai Model Organisms), aged 8 weeks, were fed with high‐fat high‐cholesterol diet (HFHC, 40% fat and 0.15% cholesterol, Cat#D12079B, Research diets). After 12‐week HFHC feeding, 1 × 10^9^ lentiviral particles encoding *villin*‐drived *Fabp2* siRNA or control siRNA (Veh) were singly administrated by tail‐vein injection. Then, the mice were killed, and aorta, small intestine and serum were collected for further analysis after another 8‐week HFHC feeding. The mice were housed in 25 ± 2°C, SPF condition. All animal experimental procedures were approved by the Animal Research and Teaching Committee at the Harbin Medical University (Harbin, China).

### 2.3 Tissue staining analysis

Whole aorta was separated and stained with Oil Red O staining solution. The aorta and small intestine were fixed in 4% paraformaldehyde and embedded in paraffin. Five µm paraffin sections were dehydrated and stained using Masson Trichrome staining kit or haematoxylin and eosin solution. For immunofluorescence staining, 10 µm aorta frozen sections were hydrated, blocked with 10% BSA solution, and incubated with anti‐moma‐2 or α‐sma antibody, then with fluorescence‐labelled secondary antibody and DAPI. The images were viewed by a fluorescence microscope (Nikon).

### 2.4 Analysis of gene expression

Total RNA was extracted from tissues by TRIZOL (Invitrogen). Complementary DNA was reversed from 500 ng RNA by using the Superscript III Reverse Transcription kit (Invitrogen), and real‐time quantitative PCR analysis was performed using SYBR Green quantitative kit (Applied Biosystems). The primer sequence for real‐time PCR was listed: *Fabp2*: F‐5′‐TAAAGTAGCCCCAACCACGA‐3′; R‐5′‐GGAACCACAGGTCTTCCAAA‐3′, *Tnf‐α*: F‐5′‐ACGGCATGGATCTCAAAGAC‐3′; R‐5′‐AGATAGCAAATCGGCTGACG‐3′, *Il‐1β*: F‐5′‐CTGGTGTGTGACGTTCCCATTA‐3′; R‐5′‐CCGACAGCACGAGGCTTT‐3′, *Mcp‐1*: F‐5′‐CCACTCACCTGCTGCTACTCA‐3′; R‐5′‐TGGTGATCCTCTTGTAGCTCTCC‐3′, *Vcam‐1*: F‐5′‐CCGGCATATACGAGTGTGAA‐3′; R‐5′‐TAGAGTGCAAGGAGTTCGGG‐3′, *Icam‐1*: F‐5′‐TTCACACTGAATGCCAGCTC‐3′; R‐5′‐GTCTGCTGAGACCCCTCTTG‐3′, *Zo‐1*: F‐5′‐CAACATACAGTGACGCTTCACA‐3′; R‐5′‐CACTATTGACGTTTCCCCACTC‐3′, *Occludin*: F‐5′‐TGAAAGTCCACCTCCTTACAGA‐3′; R‐5′‐CCGGATAAAAAGAGTACGCTGG‐3′ and *Gapdh*: F‐5′‐AGGAGCGAGACCCCACTAAC‐3′; R‐5′‐GATGACCCTTTTGGCTCCAC‐3′. Gene expression was calculated by normalizing to *Gapdh* level.

The article "Intestinal fatty acid‐binding protein mediates atherosclerotic progress through increasing intestinal inflammation and permeability" was retracted in 2022. Reasons: duplicated images; signs of a paper mill.

### 2.5 Immunoblot analysis

Total protein were extracted from small intestine, and 60 μg protein was subjected 10% SDS‐PAGE electrophoresis and electrotransferred to polyvinylidene difluoride membranes (Amersham Biosciences). The membranes were blocked in 10% BSA containing non‐fat milk, and incubated with anti‐ZO‐1, anti‐Occludin or anti‐Tubulin antibodies and relative secondary antibodies. Relative protein expression was visualized by using enhanced chemiluminescence reagents (Bio‐Rad) and quantitatively analysed by using Image J software.

### 2.6 Clinical correlation study

This study included 42 individuals, including 18 patients with carotid intima‐media thickness (IMT) ≥ 0.85 mm and 24 patients with IMT < 0.85 mm, from June 2016 to October 2018 at the Second Affiliated Hospital of Harbin Medical University. The patients with IMT < 0.85 mm were characterized by no history of angina and other heart diseases, a normal resting ECG, and normal exercise ECG stress testing. All participants have been informed clinical consent, and related analysis protocol was approved by human ethics committee of Harbin Medical University.

### 2.7 Statistical analysis

Data were represented as mean ± SEM. The Student's *t* test was used for comparing 2 groups, and anova was used for multiple groups (GraphPad). *P* < .05 was considered to be significant.

## 3 RESULTS

### 3.1 FABP2 is mainly expressed in small intestine of high‐fat high‐cholesterol diet–fed ApoE^−/−^ mice

The genetic ApoE deficiency accelerates the development of atherosclerosis in mice, especially co‐treated with western diet (high‐fat high‐cholesterol diet).^19^ Adipocyte fatty acid‐binding protein (FABP4), one member of FABP family, played a critical role in atherosclerotic process.^20^ However, whether FABP2 participated in the atherosclerotic process was unclear. To identify the potential role of FABP2 in the atherosclerotic process, we measured the distribution of FABP2 in ApoE^−/−^ mice. As shown in Figure 1A, the *Fabp2* gene was highly expressed in small intestine, as compared with in aorta, heart, kidney and visceral adipose tissue from standard chow‐fed ApoE^−/−^ mice. Furthermore, we measured the dynamic changes of intestinal *Fabp2* in HFHC‐fed ApoE^−/−^ mice. As shown in Figure 1B, HFHC diet time dependently stimulated intestinal level of *Fabp2* gene.

The article "Intestinal fatty acid‐binding protein mediates atherosclerotic progress through increasing intestinal inflammation and permeability" was retracted in 2022. Reasons: duplicated images; signs of a paper mill.

**FIGURE 1:** High‐fat high‐cholesterol diet increases the level of FABP2 in ApoE^−/−^ mice. A, The distribution of *Fabp2* in aorta, heart, kidney, visceral fat and small intestine of ApoE^−/−^ mice fed with standard chow for 12 wk. B, Male ApoE^−/−^ mice were fed with high‐fat high‐cholesterol diet (HFHC) for 0, 4, 12 and 20 wk. The *Fabp2* expression in small intestine. Data are shown as mean ± SEM (**P < .01 and ***P < .001, anova analysis was used for multiple group comparison, n = 5 mice/group)

### 3.2 Intestinal *Fabp2* knockdown attenuates HFHC diet–induced atherosclerosis in ApoE^−/−^ mice

To determine the pathophysiological role of FABP2 in atherosclerotic formation, we next specifically knockdown intestinal *Fabp2* by injecting lentiviral particles encoding *villin*‐drived *Fabp2* siRNA to HFHC diet–fed ApoE^−/−^ mice. As shown in Figure S1, lentivirus encoding *Fabp2* siRNA effectively decreased the expression levels of FABP2 protein (Figure S1A,B) and gene (Figure S1C) in ApoE^−/−^ mice, but no in aorta (Figure S1D) or visceral adipose tissue (Figure S1E). There was also no difference of body weight (Figure S1F) or fasting glucose levels (Figure S1G) between these 2 groups. Oil Red O staining of En Face aorta showed *Fabp2* siRNA significantly decreased the lipid accumulation on vascular wall, as compared with control siRNA‐treated ApoE^−/−^ mice (Figure 2A,B, *P* < .001). Furthermore, the lipid contents in aorta root were also significantly decreased in *Fabp2* siRNA‐treated ApoE^−/−^ mice (Figure 2C,D, *P* < .01). Excess immune cell infiltration was another key parameter of atherosclerosis.^21^ Figure 2E,F showed intestinal silence of *Fabp2* inhibited the infiltration of monocytes and macrophages (*P* < .001). Furthermore, *Fabp2* siRNA also suppressed the deposit of α‐smooth muscle actin and collagen (Figure 2E,G,H), which represented the vascular fibrosis. The aorta structural disorders were companied with higher levels of inflammatory cytokines, whereas *Fabp2* siRNA obviously decreased these inflammatory gene expressions (Figure 2I‐M). All these results demonstrated that intestinal silence of *Fabp2* effectively improved HFHC diet–induced atherosclerosis.

**FIGURE 2:** Blockage of FABP2 attenuates HFHC diet–induced atherosclerotic progress in ApoE^−/−^ mice. Male ApoE^−/−^ mice were fed with HFHC for 12 wk and then treated with 1 × 10^9^ lentiviral particles encoding *villin*‐drived *Fabp2* siRNA or control siRNA (Veh) for 8 wk. A‐B, Representative images of Oil Red O staining of En Face aorta (A) and quantitative analysis of relative density (B). C‐D, Oil red O staining of aorta root (C) and quantitative analysis of relative lipid deposits (D, red colour area). Scale bar = 100 μm. E‐H, Slides of aorta root were stained with moma‐2 and α‐sma antibodies, or trichrome staining solution. Representative images of staining (E), and quantitative analysis of relative density of aorta moma‐2 (F), α‐sma (G) and collagen (H). Scale bar = 50 μm. I‐M, Real‐time PCR analysis of aorta gene expression of *Tnf‐α* (I), *Il‐1β* (J), *Mcp‐1* (K), *Vcam‐1* (L) and *Icam‐1* (M). Data are shown as mean ± SEM (**P < .01 and ***P < .001, Student's *t* test was used for 2‐group comparison, n = 5‐7 mice/group)

The article "Intestinal fatty acid‐binding protein mediates atherosclerotic progress through increasing intestinal inflammation and permeability" was retracted in 2022. Reasons: duplicated images; signs of a paper mill.

### 3.3 Intestinal *Fabp2* knockdown improves intestinal permeability and inflammatory response in HFHC diet–fed ApoE^−/−^ mice

Several studies have demonstrated that gastrointestinal system affected the physiological and pathophysiological function of vascular.^5^ The abnormal intestinal permeability and subsequent endotoxin leakage into circulation might initiated vascular inflammatory response and structural disorders.^8^ In Figure S2, H&E staining of small intestine indicated HFHC diet loosed the structure of mucosa, which facilitate the leakage of toxic substances into circulation. However, treatment of *Fabp2* siRNA improved the intestinal structure (Figure 3A). Intestinal permeability was controlled by multiple epithelial tight junction protein, such as zonula occludens (ZO)‐1 and occludin.^22^, ^23^ Real‐time PCR analysis showed that silence of intestinal *Fabp2* increased the gene expression of *ZO‐1* and *occludin* (Figure 3B,C, *P* < .01). Immunoblot analysis also found the protein expression of ZO‐1 and occludin was significantly increased in *Fabp2* siRNA‐treated ApoE^−/−^ mice, as compared with control siRNA‐treated Apoe^−/−^ mice (Figure 3D‐F). The *Fabp2* siRNA treatment led to a significant reduction in the HFHC diet–induced elevation of lipopolysaccharide (LPS) level in circulation (Figure 3G), suggesting that *Fabp2* siRNA blocked LPS leakage by maintaining the intestinal structure. Next, we measured the in vivo gut permeability by oral administration of fluorescent labelled dextran (DX‐4000‐FITC).^5^ The circulating concentration of DX‐4000‐FITC was lower in *Fabp2* siRNA‐treated Apoe^−/−^ mice (Figure 3H, *P* < .01).

**FIGURE 3:** Blockage of FABP2 suppresses HFHC diet–induced intestinal permeability in ApoE^−/−^ mice. Male ApoE^−/−^ mice were fed with HFHC for 12 wk, then treated with 1 × 10^9^ lentiviral particles encoding *villin*‐drived *Fabp2* siRNA or control siRNA (Veh) for 8 wk. A, Haematoxylin and eosin staining of small intestine. Scale bar = 100 μm. B‐C, Real‐time PCR analysis of intestinal *zonula occludens (ZO)‐1* (B) and *occludin* (C) levels. D‐F, Western blot analysis of ZO‐1 and occluding (D), and quantitative analysis of relative density of ZO‐1/Tubulin (E) and occluding/Tubulin (F). G, Serum levels of lipopolysaccharides (LPS). H, The circulating concentration of DX‐4000‐FITC after mice was orally administrated with FITC‐labelled dextran. Data are shown as mean ± SEM (*P < .05, **P < .01 and ***P < .001, Student's *t* test was used for 2‐group comparison, n = 6‐7 mice/group)

Western diet has obvious effects on the gastrointestinal immune system, including infiltration of immune cells, activation of inflammatory signalling and secretion of inflammatory cytokines. To this end, we next measured the intestinal inflammatory response. Real‐time PCR results showed that administration of *Fabp2* siRNA significantly decreased the expression of inflammatory genes, including *Tnf‐α*, *Il‐1β*, *Mcp‐1*, *Vcam‐1* and *Icam‐1* (Figure 4A‐E), as compared with ApoE^−/−^ mice. Meanwhile, ELISA analysis of intestinal lysates also showed that the protein levels of inflammatory cytokines, including TNF‐α, IL‐1β and MCP‐1, were remarkably decreased in *Fabp2* siRNA‐treated ApoE^−/−^ mice. All these results demonstrated that specific intestinal knockdown of *Fabp2* effectively protected against HFHC diet–induced intestinal inflammation and permeability, which accelerated the atherosclerotic process.

The article "Intestinal fatty acid‐binding protein mediates atherosclerotic progress through increasing intestinal inflammation and permeability" was retracted in 2022. Reasons: duplicated images; signs of a paper mill.

**FIGURE 4:** Blockage of FABP2 inhibits intestinal inflammatory response in ApoE^−/−^ mice. Male ApoE^−/−^ mice were fed with HFHC for 12 wk and then treated with 1 × 10^9^ lentiviral particles encoding *villin*‐drived *Fabp2* siRNA or control siRNA (Veh) for 8 wk. A‐E, Real‐time PCR analysis of inflammatory gene expression on small intestine. F‐H, Intestinal production of TNF‐α, IL‐1β and MCP‐1. Small intestine was collected and homogenized, and the levels of cytokines TNF‐α (F), IL‐1β (G) and MCP‐1 (H) were measured by ELISA. Data are shown as mean ± SEM (*P < .05, **P < .01 and ***P < .001, Student's *t* test was used for 2‐group comparison, n = 6‐7 mice/group)

### 3.4 Circulating FABP2 is closely correlated with atherosclerotic parameters in clinical patients

Measurement of carotid intima‐media thickness (IMT) is one of gold parameters for the diagnosis of cardiovascular disease.^24^ Therefore, we recruited 18 patients with carotid intima‐media thickness (IMT) ≥ 0.85 mm and 24 patients with IMT < 0.85 mm for clinical study. As shown in Table S1, there was no difference about age, sex, fasting glucose level, insulin or HOMA‐IR between these 2 groups, but human patients with IMT < 0.85 mm had lower levels of BMI, total cholesterol and triglyceride (*P* < .05). On the contrast, *patient*s with higher IMT value had higher level of circulating FABP2 than patients with lower IMT value (Figure 5A, *P* < .01). The Pearson's correlation analysis also supported that plasma level of FABP2 was positively correlated with carotid IMT value (Figure 5B, *r* = .4517, *P* < .05). Furthermore, FABP2 was also positively correlated with atherosclerotic parameters, including total cholesterol (Figure 5C, *r* = .5034, *P* < .01) and triglyceride (Figure 5D, *r* = .5503, *P* < .01). These clinical data indicated that FABP2 was a potential diagnostic biomarker for cardiovascular diseases.

The article "Intestinal fatty acid‐binding protein mediates atherosclerotic progress through increasing intestinal inflammation and permeability" was retracted in 2022. Reasons: duplicated images; signs of a paper mill.

**FIGURE 5:** Circulating FABP2 is closely correlated with atherosclerotic parameters in clinical patients. A, The plasma FABP2 levels in 18 patients with carotid intima‐media thickness (IMT) ≥ 0.85 mm and 24 patients with IMT < 0.85 mm. B‐D, The correlation between circulating levels of FABP2 and IMT (B), total cholesterol (C) and triglyceride (D). Data are shown as mean ± SEM (**P < .01, Student's *t* test was used for 2‐group comparison, and Pearson's analysis was used for the correlation)

## 4 DISCUSSION

Therapeutic intervention of intestinal homeostasis protected against atherosclerotic process, including reduction of plaque formation and inflammatory responses.^5^, ^8^ The maintenance of gut permeability through regulating tight junction protein was the determining procedure. The disruption of gut permeability contributed to the worsen consequence of atherosclerosis. In the present study, our findings supported that the increased intestinal level of FABP2 affected the high‐fat high‐cholesterol diet–induced atherosclerosis. Special silence of intestinal *Fabp2* decreased aorta plaque formation, structural disorders and vascular inflammation. Mechanistically, knockdown of intestinal *Fabp2* inhibited western diet–induced gut permeability by up‐regulation of tight junction factors, including ZO‐1 and occludin, and suppressed intestinal inflammatory response. In clinical study, our results also identified increased plasma level of FABP2 was positively correlated with carotid intima‐media thickness (IMT) and lipid parameters, critical parameters of atherosclerosis.

The crosstalk between gastrointestinal system and cardiovascular homeostasis is emerging as a hot topic in recent years. Koeth et al^25^, reported that intestinal trimethylamine‐N‐oxide (TMAO), produced from L‐carnitine metabolism, promoted atherosclerosis in human and mice. The changes of intestinal microbiota directly or indirectly affected the development of cardiovascular diseases (CVDs). *Akkermansia Muciniphila*, one of major good microbial components, protected against western diet–induced mouse atherosclerosis.^5^ On the contrast, the intestinal component of *Citrobacter*, bad microbial bacteria, was positively associated with IMT in human patients.^26^ Moreover, TMAO could injure cardiac activation and facilitated ischaemia‐induced ventricular arrhythmia.^27^ Intestine‐derived lysophosphatidic acid (LPA) accelerated the development of atherosclerosis dependent on dyslipidaemia and inflammation.^28^ All these findings supported intestinal homeostasis could determine the consequence of western diet–induced atherosclerosis.

The article "Intestinal fatty acid‐binding protein mediates atherosclerotic progress through increasing intestinal inflammation and permeability" was retracted in 2022. Reasons: duplicated images; signs of a paper mill.

The abnormal leakage of intestinal contents, such as toxic endotoxin and bacteria, contributed to multiple of diseases. Both animal studies and clinical observations have demonstrated that the severe degree of intestinal endotoxemia was accompanied with hepatitis and cirrhosis.^29^ In patients with alcohol‐induced liver diseases, increased intestinal permeability facilitated the macromolecules and endotoxemia into circulation.^30^ Recently, several studies have demonstrated that abruption of intestinal permeability exacerbated the atherosclerotic process.^5^, ^8^ The down‐regulated expression of tight junction factors, such as ZO‐1 and occludin, was the major reason for increasing intestinal permeability.^22^, ^23^ Consistently, our study also found the transcriptional suppression of tight junction factors occurred in severe atherosclerotic mice, whereas their up‐regulation improved vascular remodelling in *Fabp2* siRNA‐treated mice.

Mechanistically, a possible explanation was specific knockdown of intestinal *Fabp2* effectively inhibited the expression of inflammatory cytokines. Amount of studies have demonstrated that excessive intestinal inflammation was one of key factors determining the biogenesis and function of epithelial zonulin proteins, and consequent the intestinal tight junction. Chronic inflammatory activation severely disrupted the tight junction integrity in multiple diseases.^10^ Nuclear factor (NF)‐κB, one of key transcriptional factors, determined the process of intestinal inflammation.^31^ Targeting inflammatory response was an effective approach to maintain intestinal biological function. Some beneficial intervention could protect against the intestinal inflammation‐induced disruption of tight junction.^11^, ^12^ Therefore, suppression of intestinal FABP2 was a potential therapeutic way to alleviate the incidence of atherosclerosis.

The article "Intestinal fatty acid‐binding protein mediates atherosclerotic progress through increasing intestinal inflammation and permeability" was retracted in 2022. Reasons: duplicated images; signs of a paper mill.

Another applicable finding was circulating level of FABP2 was significantly up‐regulated in patients with cardiovascular diseases and positively associated with IMT. Amounts of clinical studies have demonstrated that plasma FABP2 concentration was a useful biomarker of intestinal barrier homeostasis.^32^, ^33^, ^34^ Moreover, FABP2 was also a marker of Crohn's disease.^35^ However, our study firstly provided the evidence plasma FABP2 was a potential biomarker for cardiovascular disease diagnosis. Furthermore, it supported intestinal FABP2 determined the gastrointestinal homeostasis in diet‐induced atherosclerosis.

## CONFLICT OF INTEREST

The authors declare that they have no conflicts of interest.

## AUTHOR CONTRIBUTIONS

Lulu Zhang, Fan Wang and Jiajun Wang performed the experiments and analysed the data; Yongshun Wang and Yan Fang designed, discussed the study and wrote this manuscript.

## Supporting information

Figure S1

Figure S2

Table S1

## Data Availability

The data that support the findings of this study are available on request from the corresponding author. The data are not publicly available due to privacy or ethical restrictions.
